# Temporal Relation Extraction with Joint Semantic and Syntactic Attention

**DOI:** 10.1155/2022/5680971

**Published:** 2022-04-28

**Authors:** Panpan Jin, Feng Li, Xiaoyu Li, Qing Liu, Kang Liu, Haowei Ma, Pengcheng Dong, Shulin Tang

**Affiliations:** ^1^Aerospace Information Research Institute, Chinese Academy of Sciences, Beijing 100190, China; ^2^Key Laboratory of Network Information System Technology (NIST), Aerospace Information Research Institute, Chinese Academy of Sciences, Beijing 100190, China; ^3^University of Chinese Academy of Sciences, Beijing 100049, China; ^4^School of Electronic, Electrical and Communication Engineering, University of Chinese Academy of Sciences, Beijing 100190, China; ^5^QILU Research Institute, Aerospace Information Research Institute, Chinese Academy of Sciences, Jinan 250000, China; ^6^Chongqing Zhixing Hongtu Technology Co., Ltd, Chongqing 401120, China

## Abstract

Determining the temporal relationship between events has always been a challenging natural language understanding task. Previous research mainly relies on neural networks to learn effective features or artificial language features to extract temporal relationships, which usually fails when the context between two events is complex or extensive. In this paper, we propose our JSSA (Joint Semantic and Syntactic Attention) model, a method that combines both coarse-grained information from semantic level and fine-grained information from syntactic level. We utilize neighbor triples of events on syntactic dependency trees and events triple to construct syntactic attention served as clue information and prior guidance for analyzing the context information. The experiment results on TB-Dense and MATRES datasets have proved the effectiveness of our ideas.

## 1. Introduction

Temporal relation extraction is a subtask in relation extraction. The purpose is to identify the temporal relationship between two target events and then build a graph where nodes correspond to events and edges reflect temporal relations between the events.  Figure 1 illustrates an example sentence and its corresponding temporal graph. There are four events in the sentence, ***flying***, ***trying***, ***locate***, and ***stranded***. Different types of edges specify different temporal relations: solid line indicates “simultaneous,” solid line with arrow indicates “after,” and dotted line with arrow indicates “includes.”

Recognition of the temporal relationship between events has gained more researchers' attention along with the development of other natural language processing domains. As one of the most important tasks in information retrieval, it plays a crucial role in promoting many downstream natural language processing tasks such as narrative construction, text abstract, question answering, text implication, and knowledge map construction. Predicting the temporal relation is inherently challenging as it requires understanding the beginning and end times of an event. Finding the time anchors of events is necessary for determining the temporal relation types, which is also challenging even for humans. As a result, existing datasets related to this task are usually not large and have low interannotator agreements (IAA), increasing the difficulty of the development of this field.

Recently, dominant research on temporal extraction has begun to use neural networks instead of traditional feature-based approaches, without relying on a large number of manually labeled features. Meanwhile, some studies [1–4] that leverage pretraining language models, such as BERT [5] and RoBERTa [6], have shown prominent performance gain over the previous methods [7–9], benefiting from the better contextual understanding by the state-of-the-art Transformer [7] encoder. However, unlike other natural language understanding tasks, temporal extraction requires more accurate characterization of the two event mentions and the connection between them, which is pretty hard when the context is wide and complicated.

Syntactic parsing is the process of analyzing the text sentence to get the sentence structure, deepening the understanding of the context from syntactic level, which is another important perspective in addition to semantic level. There are two kinds of syntactic parsing: syntactic structure parsing aims at identifying the phrase structures in sentences and the hierarchical syntactic relationships between phrases, while syntactic dependency parsing aims at identifying the interdependence of words in a sentence. Relevant studies [10, 11] have shown great potential in dealing with many natural language understanding tasks, especially on relation extraction. However, there are still some neglected issues. The first problem is redundant information from the dependency tree which introduces noise and confusion because some less-informative dependencies are added to the later calculations. Another problem is that dependency type information is ignored, resulting in the loss of important information.

To address the above issues, we have explored further and found some intriguing results. The first discovery is that explicit event time clues make classifying temporal relation derived naturally. As shown in sentence 1 in Table 1, “Rose” happened yesterday, while “Crashed” happened today; then we could directly infer that “Rose” happened before “Crashed.” Besides, some temporal clues like the connection of the event pairs or some surrounding contexts reduce the difficulty of determining the temporal relation between the events. As shown in sentence 2, after tells the truth that rushed happened after receiving. In the above two examples, it is obvious that words highlighted in yellow are clue words that play a crucial role in determining the temporal relation types, while others are dispensable. Another discovery is that the syntactic relation label between two event mentions provides prior knowledge to help distinguish different temporal categories. In sentence 3, buildup is the nominal subject of halt and we could infer that buildup includes halt.

Therefore, based on the traditional neural network that contains coarse-grained information on semantic level, we bring a new syntactic attention mechanism to capture fine-grained information on syntactic level. Here we design the JSSA model which joints both semantic features and syntactic features to extract the temporal relations. First, we use Bi-LSTM model to capture global semantic information. Then we apply spacy to implement dependency analysis on given sentences, obtaining the syntactic relations between tokens. For event mentions, we get their neighbor triples on dependency trees as potential clue information candidates and their original syntactic relation as prior information. Finally, we apply mixed attention like the work of Peng et al. [12] to filter out the noise and capture key information which helps to determine the temporal relations between events quickly and accurately.

The main contributions of this work are summarized as follows:

1. We directly extract neighbor triples related to event mentions on syntactic dependency trees as clue information candidates, avoiding suffering from the noise in automatically generated dependency trees and reducing confusions to understand temporal relations.
2. The new feature of syntactic dependency type, which served as prior information, is incorporated into syntactic attention to help predict the temporal relation between events.
3. We propose JSSA, a model combining both semantic features as coarse-grained information and syntactic features as fine-grained information, which finally improves the performance of temporal relation extraction with good robustness.

## 2. Related Work

### 2.1. Traditional Methods

Early studies on temporal relation extraction mainly adopt rule-based models, which require a complete set of rules relying on linguistic knowledge and discrete features in the text. Allen et al. [13] introduced an interval-based temporal logic, together with a computationally effective reasoning algorithm based on constraint propagation. Passonneau et al. [14–18] focused on the expansion of rules and defined new rules based on linguistic knowledge by utilizing information such as tenses, parts of speech, rhetorical relations, expressions, and pragmatic constraints. Chambers et al. [19] proposed specifying temporal relations from a narrative event chain, which firstly extracts a series of narrative events containing common arguments from the text, identifies the temporal relations between the events, and then combines them according to the temporal sequence to form an event chain. In general, the rule-based methods have great limitations though the accuracy is satisfied, and the recall is not ideal, so it is difficult to land, and application scenarios are limited.

TimeML [20](Time Markup Language) is a set of labeling systems defined by International Organization for Standardization (ISO), whose purpose is to standardize the annotation method of time sequence information in the text. In the process of continuous improvement of the system, corpus labeling methods are gradually standardized, and a series of corpora such as TimeBank come into being. TimeBank [21] corpus is based on TimeML annotation system and is the mainstream corpus for researchers to identify temporal relationships. In addition, Chambers and Cassidy [22] adopt a mechanism of forced annotation between adjacent sentences to further process the corpus due to the sparse temporal links of the annotations in the TimeBank corpus and thus construct a higher relational density of the corpus, Timebank-Dense.

Pustejovsky et al. [21] extracted event attribute features manually marked in the corpus based on TimeBank corpus and trained the classifier with the maximum entropy algorithm to complete the recognition of temporal relations. Chambers et al. [8] subsequently proposed a two-stage classifier, in which the first stage extracts annotated features from the corpus and then extracts lexical, syntactic, and semantic information from external knowledge bases such as WordNet [23] and VerbOcean [24] to combine the two features. In the second stage, these features are used to identify temporal relationships to improve model performance further. Bethard et al. [25] regarded the time sequence relation recognition task as a paired classification task and completed the time sequence relation recognition with support vector machine model like various features based on syntax and semantics. *Mirza* et al. [26] found that simple feature sets have better performance compared with complex features using semantic role labeling and deep semantic parsing and then discussed the influence of using inverse relation and transitive closure to extract new training instances and do further study on this basis.

Machine learning has made significant progress in identifying temporal relationships of events, but temporal relationships are a global concept, not limited to event pairs. To construct a global time chain, researchers try to use a combination of machine learning and linear programming reasoning to optimize the experimental results. Chambers et al. [27] proposed a linear programming decision framework with two types of implicit global constraints to achieve global consistency and improve recognition performance. Denis et al. [28] proposed representing the event and time with the end-points of the event interval to simplify the constraint complexity and optimize on a specific subset of the whole sequence graph. Yoshikawa et al. [29, 30] utilized Markov network reasoning model to jointly identify different types of temporal relations and optimize them from sentence and discourse levels to improve temporal relationship recognition performance. Do et al. [31] put forward an article event representation method based on time interval, in which the events in a document are constructed into chains according to the event sequence, and then the global optimization of event chain is carried out by using integer linear programming and the system performance is further improved by using event codesignations. Li et al. [32] proposed a chapter-level global reasoning model to mine the temporal relationship between events at the document level, which improves the global reasoning model by using chapter-level constraints derived from event semantics. Ning et al. [33] proposed a joint reasoning framework, which utilizes the connection between timing sequence and causality to construct a variety of constraints and complete the joint identification of timing sequence and causality.

### 2.2. Neural Network Methods

Neural networks have been popular for their excellent semantic representation and self-learning capabilities in various tasks in the field of natural language processing and their superiority has been demonstrated in a number of studies. Many neural models have been proposed to capture temporal relation relations, such as the basic CNNs and LSTMs [34, 35]. Dligach et al. [34] utilized the temporal convolution neural network to learn the hidden feature representation. Ensemble models [36, 37] apply the recurrent neural model combined with SVMs and rules on clinical domain to improve performance on relevant tasks. Sorokin et al. [38] demonstrated that it is beneficial to consider other relations in the sentential context for sentence-level relation extraction, so the context representations are combined with an attention mechanism using a novel LSTM-based encoder. Tourille et al. [35] fed character vector and word vector combining with other attribute features into bidirectional LSTM model to complete the identification of inclusion relation between medical events. Leeuwenberg et al. [39] put forward a novel paradigm directly predicting start and end points for events from the text, constituting a timeline without going through the intermediate step of predicting temporal relations as in earlier work. Zhang et al. [40] proposed using the depth bidirectional LSTM model to identify the temporal sequence of events, alleviating the problem that the structure of the current neural network model is too shallow. Han et al. [1] put forward the idea that joint event and temporal relation, which is different from pipeline methods, predicts a candidate as nonevent if all temporal relations related to this candidate event are vague. By improving the accuracy of event extraction, the subsequent temporal relation task becomes easier. Han et al. [41] also proposed a deep structured learning framework, composed of a recurrent neural network and a structured support vector machine. The neural network automatically learns representations that account for long-term contexts to provide robust features for the structured model. At the same time, the SSVM incorporates domain knowledge such as transitive closure of temporal relations as constraints to make better globally consistent decisions. Besides, researchers [42] employed distributed constraints from probabilistic domain knowledge to solve the problems of biased predictions on dominant temporal relations when the training data is limited. Wang et al. [4] proposed a new framework that applies logical constraints within and across multiple temporal and subevent relations by converting these constraints into differentiable learning objectives. Mathur et al. [43] put forward a method leveraging rhetorical discourse features and temporal arguments from semantic role labels as well as local syntactic features through a Gated Relational-GCN model. Tan et al. [44] tried to embed events into hyperbolic spaces and train a classifier to capture temporal relations. Breitfeller et al. [45] developed a novel framework to explore semantic information provided by explicit textual time clues. Wen et al. [46] adopted a Stack-Propagation framework to incorporate predicted relative event time for temporal relation classification.

At the same time, syntactic analysis has been another prominent approach for predicting temporal relation. Bunescu et al. [47] presented a novel approach to relation extraction, based on the observation that the information required to assert a relationship between two named entities in the same sentence is typically captured by the shortest path between the two entities in the dependency graph. Wang et al. [48] proposed a new convolution dependency path kernel that increases the feature space by introducing bias towards more syntactically meaningful feature space. It clearly explains how different kernels are related to each other and why some are superior to others. Boella et al. [49] presented a technique that uses syntactic dependencies between terms extracted with a syntactic parser to automatically extract semantic knowledge. It transforms all the surrounding syntax of the semantic information into abstract textual representations, which are then used to create a classification model through a standard Support Vector Machine system, guaranteeing robustness when facing the length and complexity of the sentences. Gan et al. [50] put forward a novel method based on syntactic and semantic features, where the feature of dependency relation composition is obtained through the combination of the respective dependency relations between entities. The verb feature with the nearest syntactic dependency is captured from dependency relation and POS (part of speech). Zhou et al. [51] leveraged the shortest dependency path tree to generate structured dependency features, structured phrase features, and flattened dependency features. Xu et al. [52] incorporated specific dependencies between mention pairs within the standard self-attention mechanism and throughout the overall encoding stage, designing two alternative transformation modules inside each self-attention building block to produce attentive biases to regularize its attention flow adaptively.

Cheng et al. [53] firstly adopted bidirectional long short-term memory (Bi-LSTM) along dependency paths (DP) to solve the task of temporal relation extraction. Referring to Xu et al. [10], the position of the event trigger word in the dependency syntax is used to extract the shortest dependency path and characterize the association between the event and the participating objects. Using the bidirectional LSTM model, temporal relationship recognition is significantly more effective and efficient than machine learning methods without manual features and external resources. In general, it has been proved that syntactic features are compelling information on this task. Choubey et al. [54] introduced more event context information based on the shortest dependency path and used the bidirectional LSTM model to complete the task of sequential relation identification of event pairs within sentences. Ross et al. [55] utilized several BERT-based temporal dependency parser variants that significantly improve temporal dependency parsing.

Our work is related to the variants of Graph Neural Networks (GNN) [56–58], especially Graph Transformers [6, 59–61]. Unlike previous GNNs that aim to capture the context from *s* of each node within the graph, in this task, we aim to select and capture the most meaningful temporal clues for two specific event mentions from their connections within the graph as well as their surrounding contexts. Inspired by some methods [62, 63] committed to introducing prior information, we reserve the dependency type information as prior information without external knowledge. Finally, we adopt similar methods [64] to combine both semantic feature and syntactic feature. The dependency analysis for a given sentence is shown in Figure 2.

## 3. Methodology

We deal with the events in the text from the perspective of semantic features and syntactic features. First, we obtain semantic features of trigger words by BERT and Bi-LSTM that contain global information. Then we extract the neighbor triples directly related to the target events as potential clue information and events triple whose dependency type served as prior information. Then a mixed attention mechanism is applied to the triples. Finally, semantic features and syntactic features are fused to predict the temporal relation. The overall architecture of our JSSA model is shown in Figure 3.

### 3.1. Encoding Module

Given an input sentence *T*=[*t*_1_,…, *t*_*l*_,…, *t*_*r*_,…, *t*_*n*_] (which can be a single sentence or two consecutive sentences), *t*_*l*_ and *t*_*r*_ are triggers corresponding to the events; we apply the same tokenizer as BERT [5] to get all the subtokens. If a token *t*_*i*_ is split into multiple subtokens, we only keep the first one. Then we obtained the context representation *c*_*i*_ for each word *t*_*i*_ by using the pretrained BERT model, which can be expressed as

(1) $$\begin{array}{c} c_{i}=\text{BERT}\left(t_{i}\right). \end{array}$$

Here *c*_*i*_ ∈ *ℝ*^*d*_1_^ and we get the BERT embedding representations *C*=[*c*_1_,…, *c*_*l*_,…, *c*_*r*_,…*c*_*n*_].

### 3.2. Semantic Feature

To enrich the contextualized representations, each token is initialized with a one-hot part of speech (POS) tag vector *p*_*i*_ and concatenate it with BERT contextualized embeddings *c*_*i*_. In this way, we obtain the final representation *S*=[*s*_1_,…, *s*_*l*_,…, *s*_*r*_,…, *s*_*n*_], where

(2) $$\begin{array}{c} s_{i}=\left[c_{i};p_{i}\right], \end{array}$$

where *s*_*i*_ ∈ *ℝ*^*d*_1_+*d*_2_^ and then we feed the sentence into Bi-LSTM model to get hidden state sequence *H*=[*h*_1_,…, *h*_*l*_,…, *h*_*r*_,…, *h*_*n*_]. Concatenate *h*_*l*_ and *h*_*r*_(*h*_*l*_, *h*_*r*_ ∈ *ℝ*^*d*_3_^) that represent hidden states of left event and right event to get sentence-level temporal relation vector representation of trigger pairs:

(3) $$\begin{array}{c} h_{\text{triggers}}=\left[h_{l};h_{r}\right]. \end{array}$$

### 3.3. Syntactic Feature

Syntactic parsing is one of the critical technologies in natural language processing. It is the process of analyzing the input text sentence to obtain the syntactic structure of the sentence. Syntactic parsing refers to the relationship between the various components of a sentence, and it is divided into syntactic structure parsing and dependency parsing. Syntactic structure analysis is applied to obtain the syntactic structure of the whole sentence, while dependency analysis is applied to obtain the dependency relationship between words. Dependent grammar reveals its syntactic structure by analyzing the dependent relations among the components of a language unit and maintains the core verb which is the central component that governs the other components in a sentence, but it is not governed by any other components; thus all the dominated components are subordinate to the dominant in a particular dependent relationship.

Words that have a direct syntactic dependency relationship with the trigger are often helpful to judge the temporal sequence relationship such as some time adverbs. This information cannot be filtered by traditional sequence encoders, so we must use syntactic dependency tools to screen these words to assist in judgment. At the same time, the syntactic relationship between two triggers also implies a sequential relationship. For example, the relation between two words that have a subject-object relationship is unlikely to be “includes,” while parallel relationship is more likely to be “simultaneous” or “sequential.”

Attention is a major innovation in the field of NLP and has achieved great success in Transformer and BERT. Here we draw on these ideas to build our attention module to capture essential information and help us make a prediction.

Given two event mentions with a left event and a right event detected from one or two continuous sentences, we apply a public dependency parsing tool to parse each sentence into a syntactic graph and connect the graphs of the two continuous sentence with an arbitrary cross-sentence edge pointing from the preceding sentence to the following one and obtain the graph *G*=(*V*, *E*), where *v*_*l*_ and *v*_*r*_ correspond to left event and right event, respectively, in *G*. For each event node *v*_*i*_, we use *𝒩*_*i*_={(*v*_*i*_, *r*_*ij*_, *v*_*j*_)*|v*_*i*_ ∈ *V*} to denote all the neighbor triples of *v*_*i*_, respectively. Here we get *𝒩*_*l*_ and *𝒩*_*r*_.

To get the query vector, we first map the event-type-event triple into a new representation:

(4) $$\begin{array}{c} q=W_{q}\cdot t_{e}+b_{q},\\ t_{e}=W_{e}\cdot \left(c_{l}{\left\|r\right\|}_{e}c_{r}\right)+b_{e}, \end{array}$$

where ‖ denotes the concatenation operation. *c*_*l*_ ∈ *ℝ*^*d*_1_^ and *c*_*r*_ ∈ *ℝ*^*d*_1_^ are left event and right event obtained from the BERT encoder, and *r*_*e*_ ∈ *ℝ*^*d*_2_^ denotes the syntactic relation of the event pair. *W*_*q*_, *W*_*e*_, *b*_*q*_, and *b*_*e*_ are learnable parameters.

Then we apply similar linear projections to get key and value vectors. Then, for each event node *e*_*i*_, we apply similar linear projections to get key and value vectors.

(5) $$\begin{array}{c} \tilde{k_{j}}=W_{k}\cdot \tilde{t_{j}}+b_{k},\\ \tilde{v_{j}}=W_{v}\cdot \tilde{t_{j}}+b_{v},\\ \tilde{t_{j}}=W_{t}\cdot \left(c_{i}\left\|r_{ij}\right\|c_{j}\right)+b_{t}, \end{array}$$

where *c*_*i*_ ∈ *ℝ*^*d*_1_^ denotes the event triggers, *c*_*j*_ ∈ *ℝ*^*d*_1_^ denotes the word directly connected to event triggers, and *r*_*ij*_ ∈ *ℝ*^*d*_2_^ denotes the dependency type between the event pair. *W*_*k*_, *W*_*v*_, *W*_*t*_, *b*_*k*_, *b*_*v*_, and *b*_*t*_ are learnable parameters.

Then we perform multihead attention to get a new context representation:

(6) $$\begin{array}{c} h_{\text{attention}}=\sum_{\left(v_{i},r_{ij},v_{j}\right)\in N_{l}\cup N_{r}}W_{\alpha }\cdot \alpha_{j}\tilde{v_{j}},\\ \alpha_{j}=\frac{\exp\left(q{\tilde{k_{j}}}^{T}/\sqrt{d_{k}}\right)}{\sum_{\left(v_{i},r_{ij},v_{j}\right)\in N_{l}\cup N_{r}}\exp\left(q{\tilde{k_{j}}}^{T}/\sqrt{d_{k}}\right)}, \end{array}$$

where *h*_attention_ is the aggregated representation computed over all neighbor tokens of nodes *v*_*l*_ and *v*_*r*_ with 8 attention heads and *h*_attention_ ∈ *ℝ*^*d*_4_^. *α*_*j*_ is the attention score of token *v*_*j*_ over a particular event node *e*_*i*_. $\sqrt{d_{k}}$ is the scaling factor denoting the dimension size of each key vector. *W*_*α*_ is a learnable parameter.

### 3.4. Feature Fusion

Through the semantic feature extraction module, we can get the complete context information, and, through the syntactic feature extraction module, we can get some critical information to supplement the global information. Combining the information obtained from these two parts can improve the robustness and accuracy of the model. We combine the two parts as follows:

(7) $$\begin{array}{c} R=\left[h_{\text{triggers}};h_{\text{attention}}\right], \end{array}$$

where *h*_triggers_ denotes the hidden state of Bi-LSTM and *h*_attention_ denotes the attention output of triggers; thus *R* ∈ *ℝ*^2*d*_3_+*d*_4_^.

### 3.5. Relation Prediction

After getting the event representations *R*, we apply a feedforward neural network to predict their relationship.

(8) $$\begin{array}{c} y_{lr}=\text{softmax}\left(W_{r}\cdot R+b_{r}\right), \end{array}$$

where *y*_*lr*_ denotes the probabilities over all possible temporal relations between events *e*_*l*_ and *e*_*r*_.

The frequency of occurrence on different temporal relationships varies greatly, and there are many solutions [65–68] to alleviate the problem of imbalance of samples. Here we choose focal loss as our loss function, which is first put forward on object detection because an image may generate thousands of candidate locations, but only a few contain objects. The class imbalance makes training inefficient as most locations are easy negatives that contribute no valid learning signal and the easy negatives can overwhelm training, thus leading to degenerate models. Here we implement it as our target function to deal with imbalanced category distribution. The training objective is to minimize

(9) $$\begin{array}{c} L_{r}=-\sum_{i}^{N}\sum_{j}^{M}\alpha {\left(1-y_{i,j}\right)}^{\gamma }\cdot \;\log\left(y_{lr,i}\right), \end{array}$$

where *N* denotes the total number of event pairs for temporal relation prediction and *M* denotes the total number of classes. *y*_*lr*,*i*_ is a binary indicator (0 or 1) if the class label *l* is correct or not based on *y*_*lr*_. *α* and *γ* are hyperparameters.

## 4. Experiments

In this section, we introduce the two main datasets that are used for temporal relation extraction. Then we give out the hyperparameter settings and define the evaluation metrics. Finally, we provide details regarding our model implementation and ablation study.

### 4.1. Datasets

Experiments are conducted on TB-Dense and MATRES datasets. Event pairs are always annotated by their appearance order in the text; that is, given a labeled event pair (*i*, *j*), event *i* always appears prior to event *j* in the text.

TB-Dense is based on TimeBank corpus but addresses the sparse-annotation issue by promoting annotators to assign labels for each edge with a new tool. A transitive reasoner automatically infers new relations based on the latest annotations, ensuring a strongly connected graph. As for annotation guidelines, it adopts the 80% confidence rule and majority annotator agreement. Finally, TimeBank-Dense achieves greater density with 12,715 links in 36 documents compared to 6,418 links in 183 TimeBank documents. The dataset defines six relations: before, after, includes, is included, simultaneous, and vague. Relevant statistics are shown in Tables 2 and 3. The proportion of vague relation is up to 43% because of mutual vague (annotators agreement), partial vague (some annotators agreement), and no vague (annotators disagreement).

MATRES is based on TB-Dense while filtering out nonverbal events. The authors propose new multiaxis modeling to better capture the temporal structure of events with significant improvements in IAA (interannotator agreement) compared to previous work. MATRES comes up with a new multiaxis modeling method to represent the temporal structure of events that unified events belonging to different axes. Then it attempts to represent event pair using two time intervals that compare both start points and end points rather than just end points. Finally, it firstly facilitates crowdsourcing to label the dataset on the premise of labeling quality assurance through qualifying test and surviving test.

### 4.2. Settings

Following [69], all sentences are tokenized with word pieces. Our implementation is based on the PyTorch version of BERT with a 12-layer transformer, 12 attention heads, and 768-dimension hidden states. We employ Adam with *β*1  = 0.9 and *β*2  = 0.999 to fine-tune the model during the training stage. The initial learning rates along with *β* and *γ* are set to 5e-5, with a dropout rate of 0.1. The maximum input word length is 128, and we set the training batch size to 4. We set the dimension of the forward and backward hidden states representation as 200. Each dependency type is mapped into 50 dimension vectors. Equilibrium factor *α* and decay factor *γ* are set to 1 and 2, respectively, on focal loss function. We train the model for 500 epochs.

### 4.3. Evaluation Metrics

We employ Precision, Recall, and micro-F1-score as evaluating metrics. Some indicators were not mentioned in the previous paper, so we use — to represent them in Table 4 without comparison. We report average results over five runs for the same setting based on the performances on the developing set.

### 4.4. Main Results

There are plenty of ideas that have been demonstrated on the two mainstream datasets. Table 4 shows their corresponding results in contrast with ours.

TB-Dense structured [41] proposes a novel framework consisting of a recurrent neural network and a structured support vector machine, which could learn long-term contexts to ensure robustness and corporate domain knowledge to provide global consistency. Joint causal [74] firstly explores causal and temporal relations jointly from the common phenomenon that a cause usually occurs earlier than its effect. DP-LSTM [53] applies shortest dependency path methods into temporal relation extraction and achieves comparable performance without using external knowledge and manually annotated attributes of entities. Globally [70] develops a probabilistic knowledge base that provides prior knowledge in the temporal order that events usually follow from the news domain. Contextualized [71] proposes a strong baseline for neural network-based models and we use it as our baseline model.

Our Joint Semantic and Syntactic Attention model outperforms the above models on all three evaluation criteria. JSSA outperforms the DP-LSTM model using syntactic dependency trees by 7.3% on F1-score. Compared with Contextualized model, our system achieves 4.0% absolute improvement on F1 measure. The result shows that our Joint Semantic and Syntactic Attention has a superior performance.

MATRES CogCompTime [72] is a system that extracts time expressions (Timex); it normalizes them to a standard format and then extracts events on the main time axis of a story and the temporal relations between events and Timexes. Perception [73] proposes new multiaxis modeling to capture the temporal structure of events better, identifying that event end points are a major source of confusion in annotation, so it only annotates TempRels based on start points.

Similar to results on TB-Dense, our proposed model shows a great improvement on MATRES. Precision and Recall increase by 4.8% and 4.9%, respectively, compared to previous models. We get a 4.8% gap on F1-score ultimately.

Through the syntactic dependency tree, we subtly extract the critical information in the text to avoid the interference of redundant information. In addition, we can also preserve global information and enhance the robustness of the model by integrating it with the traditional LSTM model. The final results demonstrate the strength of our model and the feasibility of our idea.

### 4.5. Ablation Experiment and Interpretation

Later we conducted further ablation experiments to explore the impact of different improvements on the overall performance of the model on TB-Dense dataset. From Table 5, we can see that our model obtains stable performance by adding a semantic module to capture global information. By adding a triple attention module to capture potential clue information from connected triples, our approach further provides a 3.5% F1-score gain, demonstrating the effectiveness of syntactic dependency analysis. Later we replace triple attention with tuple attention which drops dependency type and finds some performance degradation, which confirms the significance of prior knowledge about how the words are related to each other. Our Joint Semantic and Syntactic Attention model that combines global features and local features achieves the best performance ultimately.

### 4.6. Case Study

Table 6 shows some examples we conducted by different models using the DP-LSTM model as a baseline. Tuple attention means we only use event mention and corresponding neighbor tokens without their dependency types, while triple attention includes all the above. In the first example, the DP-LSTM model can capture the right temporal relation, as can other models. Meanwhile, in the second example, previous methods mistakenly predict the temporal relation as “vague,” which is the most frequent type of six types. However, we find that buildup is the nominal subject of halt by incorporating dependency relation between buildup and halt. Therefore, our approach could infer that buildup must include halt by the dependency type “nsubj.” For the third example, Bi-LSTM model predicts the temporal relation between strangle and retreats as “before.” However, with the neighbor token “until,” our JSSA model could get the information that strangle event occurred earlier and ended later than retreats. So we classify the temporal relationship between them as “includes.” The attention heat map for this sentence is shown in Figure 4.

### 4.7. Dependency Filtering

There are dependencies between sentence components in every language, and the grammatical dependencies are different in every language. Universal Dependencies (UD) [75] is an internationally recognized framework for defining grammatical relations. There are 37 general grammatical relations in English, as shown in Table 7.

The upper part of the table follows the main organizing principles of the UD taxonomy:

  Rows correspond to functional categories in relation to the head
  Core arguments of clausal predicates
  Noncore dependents of clausal predicates
  Dependents of nominals
  Columns correspond to structural categories of the dependent
  Nominals
  Clauses
  Modifier words
  Function words

Through dependency analysis, we find that some dependencies are not helpful for judging temporal relationships; for example, articles “the” and “a” are not helpful for screening critical information. Therefore, based on the relevant grammar definition and the given task, we screened out some of the 37 kinds of dependencies that were not useful for timing judgment and conducted comparative experiments on the original dataset. The new types of dependencies are shown in Table 8, and the comparison results are shown in Table 9. It can be seen that filtering dependency types have no significant influence on the final performance, which further verified our ideas.

### 4.8. Error Analysis

Further research is done on misclassified samples to explore the error reasons. The biggest problem is imbalanced labels distribution which causes overfitting when training. Furthermore, we find that some errors may be introduced in the construction of syntactic dependency relations, which will be drawn into the subsequent attention module. For example, some dependency relation labels between event pairs are incorrect, so triple information will mislead the classification. Besides, our dependencies may be based on tokens rather than phrases, which may lose some information. The next step might be to consider introducing entity information or phrase information like ERNIE [76] did.

## 5. Conclusion and Future Work

This paper proposes a novel model, Joint Semantic and Syntactic Attention, to extract temporal relation. Based on obtaining global information by a traditional neural network, we imply syntactic attention to better capture local information. On the one hand, we use the dependency relation label between event pairs as prior information to avoid some obvious errors. On the other hand, clue tokens connected to the events act as the vital information for judgment. Combining local and global features, we obtain a robust model that could accurately extract temporal relations between event pairs. Experimental results show the effectiveness of our method.

Compared with other neural network methods, we make full use of the syntactic information of the text because the event itself contains more arguments, so the use of syntactic information can effectively screen out important information, which is also an important direction in the study of the event relationship in the text. In the future, we will further utilize the argument information of events by the syntactic parser to improve the performance of temporal relation prediction.

## Figures and Tables

**Figure 1:** An illustration of a paragraph with its partial temporal graph.

**Figure 2:** An example of dependency tree.

**Figure 3:** The overall architecture of the proposed JSSA for temporal relation extraction illustrated with an example input sentence (the two events “caught” and “missed” are highlighted in red and blue colors, respectively) and its dependency tree. The upper left part shows the semantic feature extraction and the right part shows the syntactic feature extraction.

**Figure 4:** Attention heat map for given sentence.

**Table 1:** Examples of sentences with syntactic analysis.

Sentence	Syntactic relation	Relation
The stock (*e*_1_: Rose) a bit yesterday and then (*e*_2_: Crashed) today.	$e_{1}\overset{\text{conj}}{⟶}e_{2}$	Before
He (*e*_1_: Reached) on out-of-court settlement with the German-owned firm shortly before an (*e*_2_: Employment) tribunal hearing was due to get under way.	$e_{1}\overset{\text{none}}{⟶}e_{2}$	Before
(*e*_1_: Visiting) the border town of Zarit, he later (*e*_2_: Warned) severe reprisals would follow any attacks launched at Israeli soldiers or civilians when the full troop pullout does take place.	$e_{1}\overset{advcl}{\leftarrow }e_{2}$	Includes

**Table 2:** Data statistics for TB-Dense and MATRES.

Corpora		Train	Dev	Test
TB-Dense	#Documents	22	5	9
	#Relation pairs	4032	629	1427

MATRES	#Documents	255	20	7
	#Relation pairs	13K	2.6 K	837

**Table 3:** Label distribution for TB-Dense and MATRES.

Labels	TB-Dense		MATRES	
Before	384	26.9%	417	49.8%
After	274	19.2%	266	31.8%
Includes	56	3.9%	—	—
Is included	53	3.7%	—	—
Simultaneous	22	1.5%	31	3.7%
Vague	638	44.7%	133	15.9%

**Table 4:** Comparison of different approaches.

Dataset	Model	Precision	Recall	F1-score
TB-Dense	Structured [2]	0.474	0.563	0.515
	Joint causal [33]	0.458	0.605	0.521
	DP-LSTM [53]	—	—	0.529
	Globally [70]	0.500	0.624	0.555
	Contextualized [71]	—	—	0.598

	JSSA	0.605	0.662	0.633
MATRES	CogCompTime [72]	0.616	0.725	0.666
	Perception [73]	0.660	0.723	0.690
	JSSA	0.707	0.772	0.738

**Table 5:** Ablation study on TB-Dense and MATRES.

Model (*F*1-score)	TB-Dense	MATRES
JSSA	0.633	0.738
(i) Semantic module	0.496	0.565
(ii) Syntactic attention	0.598	0.692
(iii) Dependency type	0.627	0.727

**Table 6:** Case study.

Example	Model	Prediction
Princess Anne presented the medals as the Anthem was played and thousands of spectators shouted “Arise Sir Steve!”	DP-LSTM	Before ✓
	DP-LSTM + tuple attention	Before ✓
	DP-LSTM + triple attention	Before ✓
	JSSA	Before ✓

In exchange, the buildup of U.S. forces in the region would halt	DP-LSTM	Vague
	DP-LSTM + tuple attention	Before ×
	DP-LSTM + triple attention	Includes ✓
	JSSA	Includes ✓

The combined operations are designed to isolate and strangle Iraq until it retreats from Kuwait.	DP-LSTM	Vague ×
	DP-LSTM + tuple attention	Includes ×
	DP-LSTM + triple attention	Before ×
	JSSA	Includes

**Table 7:** Universal dependencies.

	Nominals	Clauses	Modifier words	Function words
Core arguments	nsubj	csubj		
	obj	ccomp		
	iobj	xcomp		

Noncore dependents	obl	advcl	advmod	aux
	vocative		discourse	cop
	expl			mark
	dislocated			

Nominal dependents	nmod	acl	amod	det
	appos			clf
	nummod			case

Coordination	MWE	Loose	Special	Other

Conj	fixed	list	orphan	punct
cc	flat	parataxis	goeswith	root
	compound		reparandum	dep

**Table 8:** Dependency relations screened out from the Universal Dependency set.

Clausal argument relations	Description
Nsubj	Nominal subject
Csubj	Clausal subject
Obj	Object
iobj	Indirect object
Ccomp	Clausal complement
Xcomp	Open clausal complement

Nominal modifier relations	Description
nmod	Nominal modifier
Appos	Appositional modifier
Case	Prepositions, postpositions, and other case markers

Other notable relations	Description
Conj	Conjunction
cc	Coordinating conjunction

**Table 9:** Comparison of different dependency relations. F1-old shows performance on original dependency type sets, and F1-new shows performance on filtered dependency type sets.

	F1-old	F1-new
TB-Dense	0.629	0.633
MATRES	0.736	0.738

## Data Availability

The data used to support the findings of this study are available at https://github.com/qiangning/MATRES and https://github.com/qiangning/TemProb-NAACL18/tree/master/data/TBDense_gold.
